# Research on SLAM Road Sign Observation Based on Particle Filter

**DOI:** 10.1155/2022/4478978

**Published:** 2022-06-20

**Authors:** Yifan Wang, Xiaoyan Wang

**Affiliations:** School of Mechanical and Electrical Engineering, Xi'an University of Architecture and Technology, Xi'an 710055, China

## Abstract

With the development of computer hardware technology, the real-time problem of visual target tracking algorithm increasingly depends on hardware solutions. The core problem of visual target tracking is how to enhance the robustness of tracking algorithm to various complex background environments and various interference factors. Aiming at overcoming the defect that the traditional SLAM (simultaneous localization and map building) algorithm based on EKF (extended Kalman filter) has a slow repair speed for environmental interference, a Monocular SLAM_WOCPF (Monocular vision SLAM based on weight optimization combined particle filter) algorithm is proposed. The weights of all particles are reoptimized in the particle set and they are combined with the tendency of particles to degenerate and deplete. In this way, the chance of self replication of low weight particles is increased, thus increasing the diversity of the whole sample. Furthermore, the improved PF (particle filter) algorithm is applied to solve the problem of road sign observation of mobile robots, so as to expand its application scope. The results show that the mean road sign errors of the Monocular SLAM_WOCPF algorithm in two noise environments are 0.332/m and 0.441/m. The conclusion shows that the Monocular SLAM_WOCPF road sign observation method proposed in this paper can effectively improve the matching success rate of visual road signs and improve the observation quality.

## 1. Introduction

Human feeling and processing information is an important field of artificial intelligence research and application. Human perception of the external world is mainly obtained through sensory organs such as vision, touch, hearing, and smell, and about 80% of the information is obtained through visual organs [1]. When the mobile robot is running, various sensors installed on the mobile robot will sense the surrounding environment in real time; collect relevant data; and, according to this information, judge the road conditions around the mobile robot, the number and direction of pedestrians, the number and direction of mobile robots, and other information. In the process of SLAM (simultaneous localization and map building), some sensors need to be used as data measurement and acquisition tools. Computers can process image and video data by simulating human visual mechanism and accomplish tasks such as image classification and target detection and tracking, which makes the research of computer vision an important part of intelligent driving system.

With the development of robots toward intelligence, the research significance of robot autonomy is becoming more and more important [2]. Among robots, the autonomous navigation of mobile robot in unknown environment fully reflects the autonomy of robot. PF (particle filter) is a Monte Carlo method. Its basic idea is to update the robot's position distribution by using new observation data [3]. Recently, PF has become the core method to solve robot problems with higher dimensions (such as SLAM). Zhang et al. used Rao-Blackwellized PF to effectively estimate the robot path and related maps [4]. Sola et al. introduced fading factor in the process of updating covariance of unscented KF (Kalman filtering) and applied it to integrated navigation, which improved the robustness of integrated navigation system when the state changed suddenly [5]. Miao and Li put forward the resampling method to solve the problem of particle degradation, which stimulated the research upsurge of PF [6]. At present, there are still many problems to be solved in PF algorithm, such as the lack of particle diversity. EKF (extended Kalman filter) can realize the optimal estimation of nonlinear system state by observing the input and output data of the system.

The sensors of the robot should take into account various tasks as much as possible, and cameras are undoubtedly an ideal choice. With their rich information and low price, cameras have attracted more and more attention in robot positioning and mapping. The development of machine vision can be applied to the working environment that is harmful to human health or the environment with high risk [2]. On the other hand, it also improves the safety of people's lives and property and is conducive to improving people's quality of life. As the target tracking and filtering technology is widely used, it is closely related to national defense construction and people's daily life. In recent years, the research in related fields has also been paid attention to by the relevant state departments. Therefore, it has a profound realistic background to study target tracking in the field of nonlinear estimation and the application of PF in road sign observation.

## 2. Related Work

### 2.1. Development Status of Mobile Robots

SLAM problem of mobile robot includes the determination of its own pose information and the acquisition and processing of external environment information. When moving in an unknown environment, the robot uses its own sensors to calculate its own position information and detect unknown road signs around it. With the realization of industrialization and informatization in the 21st century, robot technology has been further developed and improved.

Nasir et al. get feedback information through trial and error iteration between robot and environment to optimize the strategy [7]. It does not depend on the environmental model and prior knowledge, and it has the characteristics of autonomous learning and online learning. It has gradually become the research hotspot of robot path planning in unstructured environment. Jin-Chun and Shin-Dug put forward a hierarchical learning method based on selection. In the first layer, Q-learning algorithm is used to train the basic behaviors of sports, and in the second layer, these basic behaviors are coordinated to solve the planning tasks. Simulation results show that this algorithm can be well applied to path planning in unknown environment [8]. Yun-Won et al. use Monocular RGB vision sensor to build a double-layer reinforcement learning network structure, which can achieve a good obstacle avoidance effect and lay a good foundation for the realization of path planning [9]. Silva et al. obtained the optimal parameters by optimizing the strategy parameters [10].

On the basis of Li et al.'s traditional genetic algorithm, an improved genetic algorithm is proposed, which uses serial number coding and genetic operators suitable for this coding mechanism. At the same time, more new mutation operators, insertion operators, and deletion operators are added, which improves the optimal preservation strategy, finally improves the running speed of the algorithm, and enhances the obstacle avoidance ability in the search process [11]. Jia et al. proposed an idea of RRT (rapid-exploring random tree) algorithm and rolling path planning to guide mobile robots to avoid obstacles online [12]. Sun et al. proposed a path planning method for high degree-of-freedom articulated mobile robot with fast random search tree. To realize the path planning in high-dimensional space, it first describes a robot theme selected according to the complexity of the path and then selects the robot joints involved, that is, the path planning with adaptive dimensions of configuration space and sampling [13]. Fang et al. proposed an improved path planning method for mobile robots based on the traditional bee colony algorithm. This method combines artificial bee colony algorithm as a local search process and uses evolutionary programming algorithm to refine the feasible path found by a set of local solutions, thereby improving the accuracy of the algorithm and shortening the search time [14].

### 2.2. Overview of PF Research

The core idea of PF algorithm is to use a group of particle sets with different weights to represent the prior density function, then calculate the likelihood of each particle, and finally fuse the prior value data of each particle and the newly obtained likelihood data, so as to obtain an approximate particle set that can describe the posterior density function of the estimated state.

In just a few decades, the application scope of PF has been continuously expanded, such as in the fields of economics, traffic control, wireless signal processing, and military. PF is playing a huge role.

Chen et al. solved the problem of particle degradation by adding resampling process. The basic idea of resampling is to copy the particles with high weights in the resampling stage to achieve the purpose of suppressing the increase of the number of particles with low weights [15]. A new PF algorithm of particle swarm optimization simulated annealing proposed by Zhu et al. overcomes the difficulty of sampling in high-dimensional space [16] Algorithm 1. Vallivaara et al. designed a real-time PF tracking algorithm with distributed parallel PF tracking function according to the data concurrency characteristics inside PF, which was proved to meet the time constraints of hard real-time systems [17]. Yang et al. proposed using unscented KF as a proposed distribution function for sampling particles [18]; In the related research on multitarget tracking estimation, Gil Aparicio et al. pointed out that the application of PF in multitarget tracking requires not only accurate modeling technologies such as new targets, disappearances, false alarms, false alarms, and over reporting, but also complex and variable technologies such as multisensor information fusion [19].

In the real world, people's life scenes and problems are mostly nonlinear, so linear filtering is far less widely used than nonlinear filtering. KF is the best estimation under linear Gaussian model. Moratuwage et al. argued that KF is only a special case of Bayesian filtering. Bayesian filtering provides the best research idea for state estimation of dynamic systems [20]. Do et al. combined target tracking with deep learning, applied target tracking to computer vision tracking, and expanded the application range of target tracking [21].

## 3. Research Method

### 3.1. Motion Model of Mobile Robot

The mobile robot is generally a highly nonlinear system, so it is difficult to accurately model the robot. Generally, the simplified approximate model is established. However, the error will be introduced into the approximate model, which is called model noise, and the sensor observation will also produce error, which is called observation noise. For the convenience of research, all noises are assumed to be Gaussian white noises in this paper.

There are many kinds of mobile robots, which can be divided into indoor mobile robots and outdoor mobile robots according to the working environment. Usually, the constraints can be classified into complete constraints and non-holonomic constraints. The complete constraints limit only the spatial position of the controlled object or both the spatial position and the motion speed, so they are called geometric constraints, while the non-holonomic constraints are constraints on the motion speed of the system and cannot be converted into spatial position constraints through integration. Simply put, they are non-integrable velocity constraints.

In this paper, the path tracking problem of mobile robot is described as taking an effective control decision and designing an appropriate control algorithm with the cooperation of a certain navigation system, so that the mobile robot moves in the plane rectangular coordinate system according to the curve planned beforehand, which is called the path tracking problem of mobile robot.

In the research of tracking control of mobile robots, it is generally assumed that the wheels of mobile robots touch the ground in a point way, satisfying the assumption that there is only pure rolling at the contact point [16], but no longitudinal sliding or lateral sliding. That is to say, this non-holonomic constraint is ideal, and it strictly satisfies the mathematical definition of non-holonomic constraint. If the mobile robot moves on a plane, then the rectangular coordinate system XOY can be set as the global coordinate system, as shown in Figure 1.

From Figure 1, aiming at the point *P*, the discrete kinematics model of the mobile robot can be obtained by using analytical method and coordinate operation, and its expression is as follows:

(1) $$\begin{array}{c} \left[\begin{array}{c} x_{p}\left(k+1\right)\\ y_{p}\left(k+1\right)\\ \theta_{p}\left(k+1\right) \end{array}\right]=\left[\begin{array}{c} x_{p}\left(k\right)\\ y_{p}\left(k\right)\\ \theta_{p}\left(k\right) \end{array}\right]+\Delta T\left[\begin{array}{c} \cos\;\theta_{p}\left(k\right)\\ \sin\;\theta_{p}\left(k\right)\\ 0 \end{array}\right]\left[\begin{array}{c} v_{p}\left(k\right)\\ w_{p}\left(k\right) \end{array}\right], \end{array}$$

where Δ*T* is the sampling time, the control input of the mobile robot is *u*_*p*_(*k*)=[*v*_*p*_(*k*), *w*(*k*)]^*T*^, and its state vector is *q*(*k*)=[*x*_*p*_(*k*), *y*_*p*_(*k*), *θ*_*p*_(*k*)]^*T*^.

In this module, an algorithm is designed to find the best reference signal, and the reference signal is selected as the robot's expected heading angle and the road surface curvature in front. The third module is the feedback controller, which takes the reference signal and the actual pose of the robot as the controller inputs, calculates the appropriate control quantity according to a certain control method, and sends it to the fourth module. The fourth module is the final control object mobile robot, that is, the mechanical realization part of the control quantity. For simplicity, only the wheel load of the mobile robot when it is stationary or moving in a straight line at a uniform speed is considered here. The load diagram of the driving wheel and universal wheel of the mobile robot is shown in Figure 2.

Assuming that the wheels are rigid wheels (with the elastic deformation being negligible) and the center of mass of the mobile robot is on the longitudinal axis of symmetry, according to the principle of force balance, we can obtain the vertical load on the driving wheel and the universal wheel as follows:

(2) $$\begin{array}{c} F_{f}=\frac{Mgl_{b}}{l_{a}+l_{b}},\\ F_{l}=F_{r}\frac{Mgl_{a}}{2\left(l_{a}+l_{b}\right)}. \end{array}$$

Among them, *c* is the center of mass of the mobile robot; *F*_*f*_ is the reaction force of the universal wheel on the ground; *F*_*t*_, *F*_*f*_ is the reaction to the force of the driving wheel on the ground; *M* is the total mass of the mobile robot; *l*_*a*_ is the horizontal distance from the universal wheel to the center of mass *c*; *l*_*b*_ is the horizontal distance from the axis of the two driving wheels to the center of mass *c*; and *g* is the gravitational acceleration.

Since the world coordinates of each characteristic road sign are constant, (*x*_*i*_, *y*_*i*_) is used to represent the coordinates of the *i*th characteristic road sign *B*_*i*_, and (*x*_*c*_(*k*), *y*_*c*_(*k*)) is the coordinates of the center point of the mobile robot at time *k*, so the observation model is as follows:

(3) $$\begin{array}{c} z\left(k\right)=\left[\begin{array}{c} r\left(k\right)\\ \beta \left(k\right) \end{array}\right]=\left[\begin{array}{c} \sqrt{{\left(x_{i}-x_{c}\left(k\right)\right)}^{2}+{\left(y_{i}-y_{c}\left(k\right)\right)}^{2}}\\ \tan^{-1}\frac{y_{i}-y_{c}\left(k\right)}{x_{i}-x_{c}\left(k\right)}-\phi +\frac{\pi }{2} \end{array}\right]+v\left(k\right). \end{array}$$

Similar to the state model, where the vector *v*(*k*) is the observed noise data, it is also set as a 0-vector, and its covariance is set as *R*(*k*).

### 3.2. Monocular Visual SLAM Road Sign Observation

#### 3.2.1. SLAM Model Description

The mobile robot uses the structured map information to constantly calibrate its own position to realize accurate positioning, or to realize accurate map construction when the current position is known by a high-precision hardware sensor system. Because SLAM mainly solves robot pose estimation and environmental feature location estimation, the modeling and positioning algorithms in the field of mobile robot navigation mainly adopt probability algorithm, and EKF, PF, and other methods are the most classic and commonly used online SLAM solutions.

Because EKF algorithm is unique in dealing with uncertain information, it has been in the mainstream position in the research of robot synchronous positioning and map construction. However, in recent years, in order to maintain the uncertainty between robots and features and between features, many researches have been devoted to reducing the computational scale of EKF algorithm. However, with the continuous increase of the number of environmental features, the computational resources are still inevitably exhausted. At the same time, EKF algorithm assumes that the state noise and the observation noise are uncorrelated white noise, but this assumption is very ideal, and more consideration should be given to colored noise when dealing with practical problems.

The appearance of PF algorithm solves the problem of state estimation of nonlinear and non-Gaussian systems. It helps to solve a large number of probability problems in solving SLAM problems and samples variables to approximate the probability with a large number of sampling distributions.

SLAM problem involves the estimation of its own position and the construction of external continuous environment map. In the research process, we usually use state vector *x*_*k*_ to represent the posture state vector of mobile robot at *k* time, *m*_*j*_ to represent the position state vector of the *j*th environmental characteristic road sign, *u*_*k*_ to represent the input control quantity exerted on the robot at *k* time, and *z*_*k*_ to represent the observation of the sensor equipped by the robot at *k* time.

Based on the Bayesian formula and the motion process of robot being Markov process, *p*(*x*_*k*_, *m|z*_1*k*_, *u*_1*k*_) can be simplified into the following formula:

(4) $$\begin{array}{c} p\left(x_{k},m|z_{1k},u_{1k}\right)\propto p\left(z_{k}|x_{k},m\right)\int p\left(x_{k}|x_{k-1},u_{k}\right)p\left(x_{k-1},m|z_{1k-1},u_{1k-1}\right)dx_{k-1}. \end{array}$$

The general model of SLAM problem can be obtained from (4).

#### 3.2.2. Road Sign Observation Realization

PF is a recursive Bayesian filtering algorithm based on Monte Carlo thought [11]. Based on the theorem of large numbers in probability and statistics theory, this method uses computer simulation technology to solve some problems that are difficult to solve directly. Monte Carlo methods randomly simulate a certain distribution through a series of sampling points. On the basis of a large number of experiments, the probability of random events is infinitely close to the frequency (Algorithm 1).

The basic idea of PF is to estimate *p*(*x*_*t*_*|z*_*t*_, *u*_*t*_) with some samples or particles {*x*_*t*_^(*i*)^}. *x*_*t*_^(*i*)^ is the *i*th sample among *M* samples, and *M* is the size of PF.

After repeating the above process several times, except for one or a few particles, the weight of other particles is approximately zero. This phenomenon is called particle degradation, and it is also an obvious problem in sequence importance sampling. It wastes a lot of computing resources on most particles whose contribution to state estimation is almost zero. Through the analysis, it can be seen that with the iterative operation of the filtering process, the variance of particle weight will increase continuously.

PF can be used in any state space description system. Its core lies in constructing a posterior probability density function, which needs to reflect the real probability distribution. By sampling the constructed posterior probability function, we can approximate the sampling process from the real distribution [13].

Let {*x*_0:*k*_^*i*^, *w*_*k*_^*i*^}_*i*=1_^*N*^ be the particles sampled from the posterior probability density function and their corresponding weights, and the weights of the particles satisfy ∑_*i*_*w*_*k*_^*i*^=1. With the above-mentioned series of particle pairs, the posterior probability density of the system can be expressed by the following formula:

(5) $$\begin{array}{c} p\left(X_{k}|Z_{k}\right)\approx \sum_{i=1}^{N}w_{k}^{i}\delta \left(X_{k}-X_{k}^{i}\right). \end{array}$$

In the formula, the solution process of posterior probability density function is transformed from integral to algebraic summation problem, and the calculation process is simplified. Take solving the statistics of function *f*(*x*) as an example, and the following formula is its expected expression:

(6) $$\begin{array}{c} E\left(f\left(x\right)\right)=\int f\left(x\right)p\left(X_{k}|Z_{k}\right)dx=\sum_{i=1}^{N}w_{k}^{i}f\left(x_{k}^{i}\right). \end{array}$$

PF tracking is a robust visual target tracking algorithm, which can effectively solve the problems of nonlinear state and non-Gaussian noise distribution in visual target tracking and can simultaneously track various state changes of visual target, without any requirement for the motion state of visual platform, and it has achieved good results in practical application. With the in-depth study of PF tracking, effectively solving these problems is of great significance to further improve the robustness of PF tracking algorithm and expand its application scope.

In order to reduce the loss of low-weight particles in each filtering, this section introduces a new algorithm, Monocular SLAM_WOCPF (Monocular vision SLAM based on weight optimization combined particle filter) algorithm.

The basic idea is to first calculate the particle swarm weight {*w*_*k*_^*i*^, *i*=0, ⋯, *N*} through important weights; then take the average value ${\bar{w}}_{k}$ of the particle swarm weight; then carry out appropriate optimization and combination operation on ${\bar{w}}_{k},w_{k}^{\prime }$${\bar{w}}_{k},w_{k}^{\prime }$; and then get a new particle set {*x*_*k*_^*i*^, *ψ*_*k*_^*i*^}_*i*=1_^*N*^.

The specific formula is as follows:

(7) $$\begin{array}{c} {\bar{w}}_{k}=\frac{\sum_{i=1}^{N}w_{k}^{i}}{N},\\ \psi_{k}^{i}=\frac{K-1}{K}w_{k}^{i}+\frac{{\bar{w}}_{k}}{K}, \end{array}$$

where *K*(1 ≤ *K* ≤ +*∞*) is the scaling factor. Under the effect of weight optimization and combination algorithm, the weight of the original low-weight particles is improved, so that more particles participate in the reproduction in the resampling process.

Under the condition of camera motion, the influence of camera translation on motion detection should usually be considered. Some methods first achieve the registration of consecutive images by motion estimation and then detect the motion by frame difference or optical flow [19]. In this work, the visual saliency map based on dynamic features is regarded as a global suggested distribution for PF tracking. For simplicity, this work uses frame difference method to detect the motion in the scene as MSM (Motion Saliency Map).

(8) $$\begin{array}{c} \text{MSM}=\left|I_{k}-I_{k-1}\right|, \end{array}$$

where *I*_*k*_ represents the image at the *k* time.

Set *S*_*t*−1_, robot control quantity *u*_*t*_, and observation quantity *z*_*t*_ are used to find set *S*_*t*_. Firstly, each particle in the set *S*_*t*−1_ is used to generate an estimate of the pose of the robot at time *t*:

(9) $$\begin{array}{c} s_{t}^{\left(i\right)}∼p\left(s_{t}|u_{t},s_{t-1}^{\left(i\right)}\right). \end{array}$$

The weights required for resampling the robot path particles are calculated as follows:

(10) $$\begin{array}{c} w_{t}^{\left(i\right)}\propto \frac{p\left(s^{t,\left(i\right)}|z^{t},u^{t},n^{t}\right)}{p\left(s^{t,\left(i\right)}|z^{t-1},u^{t},n^{t-1}\right)}. \end{array}$$

In this paper, we need to match the road sign information detected at the current moment with the road sign information in the state vector according to the feature matching algorithm, so as to determine the stable and repeatable road sign points existing at the current moment. That is, each iteration only needs to extract one data item from the observation data set.

Map feature estimation is represented by {*u*^1^, *p*^1^, ⋯, *u*^*M*^, *p*^*M*^}. *u*^*i*^, *p*^*i*^ represent the Gaussian mean and variance of the *i*th map feature, respectively. When the robot is moving, if a landmark feature in the map is detected at a certain moment, the following formula is adopted to update the feature. If no new landmark feature is detected, the mean and variance are equal to the values of the previous moment.

(11) $$\begin{array}{c} u_{k+1}^{i}=u_{k}^{i}+K_{k+1}^{i}\left[z_{k+1}^{i}-h\left(u_{k}^{i}\right)\right],\\ p_{k+1}^{i}=p_{k}^{i}+K_{k+1}^{i}S_{k+1}^{i}{\left(K_{k+1}^{i}\right)}^{T}. \end{array}$$

To facilitate understanding, Figure 3 shows the algorithm flow of Monocular SLAM_WOCPF.

The implementation process of the algorithm is as follows:

1. Initialize. Determine the initial state value and covariance matrix of the mobile robot system, and sample the first 10 samples from the initial distribution.
2. Forecast. Based on the motion model of the robot, the pose of the robot at *k*+1 time is predicted by the control input.
3. Data association. The observed value at *k*+1 time is obtained and correlated with the estimated observed value of each particle at the time. These correlation processes are independent of each other.
4. Get the suggested distribution. Based on the observed values of each particle, the mean and variance of each particle's pose estimation are calculated, and a Gaussian distribution function is constructed with the mean and variance as the importance probability density function to be calculated.
5. Robot path estimation. The algorithm estimates the path of the robot and calculates the particle set used to characterize the posterior probability distribution of the robot at *k*+1 time.

## 4. Result Analysis

Under the Matlab simulation environment, the motion and observation of the mobile robot are simulated by using the above-mentioned motion model and observation model, and the simulation of the mobile robot Monocular SLAM_WOCPF is realized.

The output of KF is represented by *y*_*e*_. Both process excitation noise *β* and measurement noise *γ* are bounded, their values can only be within a certain range, and they are independent of each other. By combining iterative learning control with KF, KF iterative learning control system can give full play to the advantages of iterative learning control.

In practical engineering applications, the system can be stabilized with fewer iterations, which is conducive to improving the real-time performance of the control system. However, if the algorithm converges slowly, it will not only fail to achieve the real-time control of the system, but also affect the tracking accuracy, so it is very unfavorable for the real-time tracking control of mobile robot. The number of iterations is set to 20, the sampling time is 0.002 s, and the given time for each iteration is 2 s. The simulation results are shown in Figure 4.

It can be seen that the control system can stabilize quickly, and the tracking error is small. Therefore, it can be inferred that after adding KF, although there are interference terms *β* and noise terms *γ*, the control performance of the system does not deteriorate. In practical applications, KF has been widely used in various practical systems, which is of great significance to improve the control system's resistance to external disturbances.

For any input, the fuzzy controller should give appropriate control output, which is called completeness. The requirement of fuzzy control completeness for rule base is that at least one applicable rule should be ensured for any input. From the analysis of kinematics model, it is concluded that there is a coupling relationship between the velocity and angular velocity of the mobile robot.

The reason why the speed of the mobile robot is affected by the difference of heading angle and the bending degree of the road ahead is that, in the final analysis, the mechanical constraint of angular velocity should be considered. The tracking effect diagram in Figure 5 and the error diagram in Figure 6 can be obtained by simulating the described model.

It can be seen that the tracking error of the algorithm used in this paper is reduced, which is closer to the real state value. The reason is that the basic PF algorithm resamples to reduce the number of effective particles, and the particles selected by resampling are highly concentrated on a few heavyweight particles.

This optimization process ensures the diversity of particle population and changes the PF algorithm's practice of directly discarding low-weight particles. At the same time, in the process of moving to the best individual, the decrease of the distance between individuals leads to the increase of relative attraction. In this paper, the improved algorithm introduces a decreasing function to guide the movement of individuals, so as to avoid falling into the situation of inability to converge.

The increase of the number of particles will make up for the lack of diversity of particles to a certain extent, making very small or even almost no improvement in the accuracy of the improved algorithm after the number of particles reaches a certain level. In addition, for the same algorithm, the increase of particle number will increase the viscosity of the algorithm. To compare the simulation results more intuitively, Table 1 and Figure 7 list the average execution time of each algorithm and RMSE (Root Mean Squared Error) average in digital form.

It can be seen intuitively that the accuracy of Monocular SLAM_WOCPF algorithm is better than that of EKF_SLAM algorithm under the same particle number and the algorithm complexity is equivalent. With the increase of the number of particles, the increasing trend of precision slows down.

There are two reasons for this phenomenon: one is that PF algorithm itself has the characteristic that the accuracy changes gently after the number of particles reaches a certain level; the other is that the increase of the number of particles makes up for the deficiency of the diversity of particles, which makes more particles participate in the replication and estimation, which directly leads to weakening the weight optimization combination effect.

Therefore, the Monocular SLAM_WOCPF algorithm can increase the diversity of particle sets, delay the process of particle depletion, and slightly improve the estimation accuracy without affecting the computational complexity.

Simulating the characteristics of human visual tracking, the visual saliency area is defined as the global recommendation distribution of PF, and it is organically combined with the local recommendation distribution. When the target is caught up, the target is tracked in the local recommendation distribution, and when the target is lost, the target is searched in the global recommendation distribution. In the experiment, this tracking algorithm is compared with PF tracking, Kalman PF tracking, and unscented PF tracking. The results show that the tracking algorithm proposed in this paper not only inherits the superior local tracking ability of the traditional PF, but also can search and locate the target in the global scope as quickly as people, thus adapting to the rapid movement and large-scale transfer of the target.

In order to make the above statement more convincing, we compare the robot estimation errors of the EKF-SLAM algorithm, the algorithm in [14], and the Monocular SLAM_WOCPF algorithm. The results are shown in Figure 8.

It is not difficult to find that the estimation error of the Monocular SLAM_WOCPF algorithm is obviously lower than that of the EKF-SLAM algorithm and not higher than that of [14] algorithm. Therefore, the accuracy of Monocular SLAM_WOCPF algorithm in robot pose positioning and map building is obviously higher than that of EKF-SLAM algorithm, and its pose positioning accuracy is obviously higher than that of [14]. The Monocular SLAM_WOCPF algorithm is practical and effective.

In order to avoid the randomness caused by noise, the noise environment is changed now. The EKF-SLAM algorithm, the algorithm in [14], and the Monocular SLAM_WOCPF algorithm are carried out in two different observation noise environments, and the process noise is the same as *σ*_*v*_=0.2 m/s, *σ*_*G*_=4°. Every simulation is conducted with 20 Monte Carlo experiments, and the results are shown in Table 2.

It can be seen that in any noise environment, the accuracy of pose estimation of Monocular SLAM_WOCPF algorithm is the best compared with the other two algorithms, and the average road sign errors of the Monocular SLAM_WOCPF algorithm in the two noise environments are 0.332/m and 0.441/m, respectively, which are obviously less than those of the other algorithms.

Fundamentally, this is because the weight optimization combination introduced in Monocular SLAM_WOCPF can improve the particle distribution; the rotation factor and movement factor can make the particle set approach the real robot pose state more quickly; and at the same time, rotation factor and movement factor can improve the problem of particle degradation and dilution in the algorithm, making the estimation result more stable and accurate.

Given the initial pose and expected path of the mobile robot, if the initial position is outside the trackable area of the expected path, a temporary path needs to be planned first, and the whole path formed by the connection of the temporary path and the expected path is regarded as the track to be tracked by the mobile robot. Clamping slots are arranged at the sides of both ends of the load adjustable layer to realize the longitudinal position adjustment of the weight block, and the weight block can also realize the lateral position adjustment through the clamping slots on the baffle. Therefore, that lay can adjust the position of the weight block in a large range on a two-dimensional plane. In addition, it can be changed by adjusting the height of the aluminum alloy support column between the robot chassis and the load adjustable layer.

Once all the states reach the sliding mode surface, the system will no longer be sensitive to parameter changes and external disturbances and only keep moving in the sliding mode. By combining the moment calculation method with the adaptive method, we can make full use of the known information of the mobile robot, thus improving the control performance of the system. However, the method of calculating moment has great dependence on the accuracy of the dynamic model of mobile robot. With the expanding application range of mobile robots, the working environment and tasks of mobile robots will become more complicated. It is necessary to consider how to extend the path planning of a single robot to the path planning of multiple robots. In addition, future robots may have to perform other tasks while planning their paths.

## 5. Conclusion

Visual target tracking is an important research direction in the field of computer vision, and robustness is the premise of practical application of visual target tracking algorithm. PF is a new filtering estimation algorithm which is widely used in nonlinear and non-Gaussian random systems. Compared with other nonlinear filtering algorithms, it is more practical. In this paper, an improved algorithm based on the traditional EKF-SLAM algorithm is proposed. Through the observation of the characteristic road signs by the mobile robot at the previous moment, combined with the system input, the position of these road signs relative to the robot at the next moment is predicted. The SLAM simulation experiment proves that the Monocular SLAM_WOCPF algorithm has the best estimation accuracy for robot pose and signpost characteristics compared with other algorithms under the same noise condition.

## Figures and Tables

**Figure 1:** Motion diagram of mobile robot.

**Figure 2:** Schematic diagram of wheel load.

**Figure 3:** The flowchart of Monocular SLAM_WOCPF algorithm.

**Figure 4:** The change of position and angle tracking error with iteration number based on KF.

**Figure 5:** Tracking effect comparison.

**Figure 6:** Error distribution comparison.

**Figure 7:** Comparison curve of simulation results of two algorithms.

**Figure 8:** Road sign estimation error.

**Algorithm 1:** Algorithm 1 PF algorithm.

**Table 1:** Statistical comparison of simulation results of two algorithms.

Algorithm	Particle number	Average execution time (s)	Estimated path RMSE average (m)	Estimate RMSE average of map (m)
EKF_SLAM	10	50.21	2.0367	2.8814
	20	123.36	1.5531	2.2417
	30	233.68	1.2347	1.8249
	40	268.7	1.0326	1.6271

Monocular SLAM_WOCPF	10	51.03	1.8824	2.6035
	20	124.66	1.4023	2.0513
	30	235.08	1.1827	1.7322
	40	265.19	1.0138	1.4369

**Table 2:** Estimation accuracy of each algorithm in two noisy environments.

Algorithm	*σ*_*r*_=0.2 m/s, *σ*_*θ*_=2°		*σ*_*r*_=0.4 m/s, *σ*_*θ*_=4°	
	Mean pose error (m)	Mean road sign error (m)	Mean pose error (m)	Mean road sign error (m)
EKF_SLAM	0.436	0.374	0.589	0.501
Reference [14]	0.723	0.445	0.869	0.664
Fast Monocular SLAM_WOCPF	0.174	0.332	0.208	0.441

## Data Availability

The dataset can be accessed upon request.
